The article "Effect of Psychological Intervention Combined with Dietary Guidance on Quality of Life and Long-Term Efficacy of Bushen Quyu Decoction in Treatment of Patients with Advanced Ovarian Cancer" was published in 2021. Journal: Evid Based Complement Alternat Med.

# Effect of Psychological Intervention Combined with Dietary Guidance on Quality of Life and Long-Term Efficacy of Bushen Quyu Decoction in Treatment of Patients with Advanced Ovarian Cancer

**DOI:** 10.1155/2021/1075513

**Published:** 2021-10-25

**Authors:** Dan Liu, Guangwen Shi, Chao Yin, Zhendong Liu, Aixia Yang

**Affiliations:** ^1^Outpatient Department, Shaoxing Central Hospital, The Central Hospital Affiliated to Shaoxing University, Shaoxing 312030, China; ^2^Department of Health Management Center, Zhangqiu District People's Hospital, Jinan 250200, China; ^3^Department of Obstetrics, Affiliated Qingdao Central Hospital, Qingdao University, Qingdao 266000, China; ^4^Department of General Medicine, Shaoxing Central Hospital, The Central Hospital Affiliated to Shaoxing University, Shaoxing 312030, China

## Abstract

**Objective:**

To study the effects of psychological intervention combined with dietary guidance on the quality of life and long-term efficacy of Bushen Quyu Decoction in the treatment of patients with advanced ovarian cancer.

**Methods:**

220 patients with advanced (stages III to IV) ovarian cancer in our hospital from May 2015 to October 2018 were selected and randomly divided into a control group and an observation group, with 110 cases in each group. The patients in the control group received basic nursing care and treatment with Bushen Quyu Decoction, and the patients in the observation group were combined with psychological intervention and dietary guidance on the basis of the treatment of the patients in the control group. The clinical efficacy, nursing satisfaction, treatment compliance, quality of life, negative emotion comparison, and long-term efficacy of the two groups were compared. Moreover, the changes of immune function indexes and the content of tumor markers were compared between the two groups.

**Results:**

The total effective rate of treatment in the observation group (64.55%) was higher than that in the control group (31.82%). The nursing satisfaction of the observation group was 94.55%, the nursing satisfaction of the control group was 84.55%, and the difference was statistically significant (*p* < 0.01). The treatment compliance of the observation group was 98.18%, the treatment compliance of the control group was 82.73%, and the difference was statistically significant (*p* < 0.0001). After nursing, the Anxiety Self-Rating Scale (SAS) score and Self-Rating Depression Scale (SDS) score of the two groups of patients were decreased (*∗p* < 0.05), and the score of the observation group decreased more significantly (^Δ^*p* < 0.05). After nursing, the scores of the two groups of patients in social/family status, physical function, physiological function, and emotional status increased (*∗p* < 0.05), and the observation group was significantly higher than the control group (^Δ^*p* < 0.05). After nursing, the CD3+, CD4+, CD4+/CD8+ levels of the observation group were significantly higher than the control group (*p* < 0.05). The CD8+ level of the observation group was significantly lower than the control group (*p* < 0.05). After nursing, the levels of tumor markers in the two groups were decreased (*∗p* < 0.05), and the observation group was downregulated more significantly than the control group (^Δ^*p* < 0.05). The two-year cumulative survival rate of the observation group was 78.18%, and the two-year cumulative survival rate of the control group was 54.55%. The observation group was significantly higher than the control group (*p* < 0.05).

**Conclusions:**

Psychological intervention combined with dietary guidance can significantly improve the quality of life and mental state of patients with advanced ovarian cancer, enhance the patient's immune function, reduce the serum tumor markers carcinoembryonic antigen (CEA) and carbohydrate antigen (CA199) levels, and improve survival rate and survival time, which has important clinical significance.

## 1. Introduction

Ovarian cancer is one of the common gynecological malignancies in clinic with high morbidity and mortality [1]. In recent years, the incidence of ovarian cancer in young women has been increasing year by year, and it is the fifth leading cause of cancer-related death in women worldwide and also the main cause of death of gynecological malignant tumors, attracting more and more social attention [2]. Ovarian cancer has no obvious clinical symptoms in the early stage and is easily ignored by patients. As time goes by and the condition deteriorates, it is often in the middle and late stages when diagnosed. Advanced ovarian cancer is prone to spread and metastasis, which seriously threatens the health and life safety of women [3]. So far, the most effective way to treat advanced ovarian cancer is chemotherapy, which can inhibit the growth and spread of tumor cells through the pharmacological effects of chemotherapeutic drugs. However, chemotherapy takes a long time, and the process is more painful, which will bring health to the patient. The double burden of economy affects the physical and mental health of patients and is not conducive to the recovery of patients [4, 5]. In recent years, Chinese medicine adjuvant therapy has been widely used in the clinical treatment of ovarian cancer. By regulating the immune function of the body, it can improve the toxic and side effects caused by chemotherapy, thus inhibiting the metastasis and recurrence of cancer cells, improving the clinical efficacy, and prolonging the survival time [6, 7]. Clinical experience has shown that most patients with ovarian cancer will have different degrees of psychological problems, such as anxiety, anger, depression, giving up, and other psychological changes, so it is very necessary to implement appropriate psychological care interventions for patients [8]. Malnutrition in patients with ovarian cancer can also lead to an increase in their mortality, which can be corrected by standardized nutritional therapy [9]. Therefore, the continuous psychological intervention and the formulation of a reasonable diet plan for the patients can help improve the patients' negative psychological mood, increase the patients' confidence and courage to treat the disease, so as to improve the clinical efficacy, improve the patient's quality of life, and prolong the patient's survival time. In this study, 220 patients with advanced ovarian cancer treated in our hospital from May 2015 to October 2018 were selected as the research objects, aiming to explore the effects of psychological intervention combined with dietary guidance on the quality of life and long-term efficacy of Bushen Quyu Prescription in the treatment of advanced ovarian cancer patients. The report is as follows.

## 2. Materials and Methods

### 2.1. General Information

220 cases of advanced ovarian cancer patients treated in our hospital from May 2015 to October 2018 were randomly divided into the control group and observation group, each with 110 cases. Control group included 34 to 70 years old, average (55.23 ± 7.14) cases; clinical stage included 68 cases of stage III and 42 cases of stage IV; tumor type included 12 cases of undifferentiated carcinoma, 41 cases of mucinous carcinoma, 9 cases of embryonic carcinoma, 14 cases of granular carcinoma, and 34 cases of serous carcinoma; observation group included 33–72-year-old cases; clinical stage included 65 cases of stage III and 45 cases of stage IV; tumor types included 14 cases of undifferentiated carcinoma, 37 cases of mucinous carcinoma, 11 cases of embryonic carcinoma, 13 cases of granular carcinoma, and 35 cases of serous carcinoma. Inclusion criteria were as follows: all patients who were diagnosed by pathological diagnosis and met the diagnostic criteria in the “Guidelines for the Diagnosis and Treatment of Ovarian Malignant Tumors” [10] and patients ≥18 years old and able to communicate normally; the survival time of patients was predicted to exceed 6 months. Those who were treated for the first time were also included. Exclusion criteria were as follows: patients with heart damage or liver and kidney abnormalities; patients with mental disorders, mental disorders, or loss of consciousness; patients with other types of malignant diseases; and women in pregnancy and lactation. There was no statistically significant difference between the two groups of patients in general information, such as age, tumor type, and clinical stage (*p* > 0.05), and they were comparable. The research goals and procedures of this study have been clarified by patients and their families, and they have voluntarily signed an informed consent form, which has been approved and supported by the medical ethics committee of Affiliated Hospital of Shaoxing University (Approval No. 20150112-3).

### 2.2. Treatment Method

Patients in the control group were treated with conventional nursing and Bushen Quyu Decoction, and the observation group was treated with psychological intervention and dietary guidance on the basis of the control group.

Recipe for invigorating the kidney and removing blood stasis was as follows: *Astragalus* 25 g, Taizishen 20 g, Shan Ci mushroom 10 g, *Scutellaria barbata* 20 g, *Ligustrum lucidum* 15 g, *Codonopsis* 20 g, *Polygonatum* 15 g, *Atractylodes macrocephala* 20 g, Poria 20 g, chicken internal gold 10 g, and Scrophulariaceae 20 g. Decoction and extract were about 300 ml of juice, 1 dose/d, divided into two warm doses in the morning and evening, 4 weeks as a course of treatment, and two consecutive courses of treatment.

Psychological nursing methods were as follows. Nursing staff in the observation group took the initiative to communicate with patients and their families patiently before treatment, understand the patients' condition, personality, psychology, family situation, disease cognition, and other conditions, and listen to their feelings carefully, popularize the knowledge of ovarian cancer-related diseases for patients, improve their understanding of ovarian cancer, eliminate the doubts of patients and their families, pay attention to the patient's emotional changes and psychological state, inform the patient in advance of the possible adverse reactions during the treatment, and avoid causing the patient's emotional fluctuations, actively communicate with patients, avoid talking about sensitive topics, encourage patients to express their feelings, and listen to them patiently and comfort them, so that they can feel the care and attention of medical staff, so as to improve the compliance of patients with treatment. Family members of patients should strengthen emotional support, so that patients can feel the support and care from family members, relieve anxiety and depression, and illustrate the positive effect of a good attitude on the recovery of the disease. Besides, regular lectures on successful cases should be held to encourage patients to build up their confidence and determination to overcome the disease.

Diet care method was as follows. According to the characteristics of the patient's condition and their own conditions, the observation group was made a personalized diet plan. The patients were instructed to maintain a light diet, ate more high-fiber, high-vitamin, low-fat, and low-salt foods, and ate more fruits and vegetables during bed rest, avoided irritating foods, avoided tobacco and alcohol, and avoided intake of foods that are too high in sugar or fat. The dietary principle was to eat small and frequent meals, chew slowly, and avoided overeating.

### 2.3. Observation Index

(1) We compare the clinical efficacy of the two groups. According to the relevant content in “Evaluation Criteria for Treatment Efficacy of Solid Tumors-RECIST” [11], the efficacy is determined 4 weeks after the end of treatment. Regarding complete remission, the tumor continues to disappear for ≥4 weeks or completely disappear; for partial remission, tumor shrinkage was >70%; for stable cases, tumor shrinkage was 30% to 70%; for progression, after treatment, the extent of the lesion cannot be controlled, and the increase was > 20% or new lesions. The total effective rate of treatment (%) = (complete remission + partial remission)/total number of cases × 100%. (2) We compare the nursing satisfaction and treatment compliance of the two groups. A satisfaction survey questionnaire was used to evaluate the patient's satisfaction with the nursing staff's service attitude, operational skills, and humanistic care. The full score is 100 points: 90 points or more are considered very satisfactory, 70–90 points are considered relatively satisfactory, and less than 70 points are considered dissatisfied. The full score for compliance is 100 points: 90 points or more are full compliance, 70–90 points were for partial compliance, which refers to patients' incomprehension and resistance to some treatments and nursing procedures, and noncompliance was below 70 points, which refers to patients' serious resistance and noncompliance. (3) We compare the negative emotional state of the two groups of patients before and after intervention and using the anxiety self-rating scale and depression self-rating scale to evaluate [12]. The SAS is a self-rating scale used to evaluate the anxiety of patients. It has 20 items and is scored in reverse from 4 to 1 point. The higher the score, the higher the degree of anxiety. The 20 items of the SDS are scored on a scale of 1 to 4. The higher the score, the deeper the depression. (4) We compare the quality of life of the two groups of patients. The ovarian cancer specific scale (Functional Assessment of Cancer TherapyOvarycancerV4.0, FACT-OV4) was used to evaluate the quality of life [13], including social/family status, emotional status, functional status, and physiological status. The higher the score, the better the quality of life. (5) We compare the long-term efficacy of the two groups of patients. The follow-up was 2 years, the follow-up frequency was 2 months, the patient's survival time was recorded, and the two-year cumulative survival rate was calculated. (6) We compare the levels of T cell subsets of the two groups of patients after treatment. (7) We compare the changes of tumor markers in the two groups before and after treatment. 5 ml of fasting cubital venous blood was collected from the patient and then centrifuged at a radius of 12.5 cm, 3 000 r/min for 10 min. The flow cytometry fluorescent antibody alkaline phosphatase staining method was used to detect T lymphocyte subsets (CD3+, CD4+, CD8+, and CD4+/CD8+ cell ratio) levels, and ELISA method was used to detect tumor markers, including CEA and CA199.

### 2.4. Statistical Method

All statistical data are analyzed using SPSS23.0 statistical software (IBM, NY, USA) at least three times. Measurement data are expressed as mean ± standard deviation (SD), using *t*-test. Counting data are expressed as rate [n (%)], using *χ*^2^ test. *p* < 0.05 was evaluated as statistically significant.

## 3. Results

### 3.1. Comparison of the Clinical Efficacy between the Two Groups of Patients

As shown in Table 1, the total effective rate (64.55%) in the observation group after treatment was higher, than that of total effective rate in the control group (31.82%) (*p* < 0.001), indicating that the clinical efficacy of the observation group is better.

### 3.2. Comparison of Nursing Satisfaction and Patient Treatment Compliance between the Two Groups

The nursing satisfaction of the observation group was 94.55%, and that of the control group was 84.55%; the difference was statistically significant (*p* < 0.01)**(**Table 2**)**. The treatment compliance of the observation group was 98.18%, and the treatment compliance of the control group was 82.73%; the difference was statistically significant (*p* < 0.001) (Table 3).

### 3.3. Comparison of the Immune Function of the Two Groups of Patients after Nursing

After nursing, the CD3+, CD4+, and CD4+/CD8+ levels of the observation group were 73.04 ± 7.63, 33.25 ± 6.31, and 1.52 ± 0.31, which were significantly higher than those of the control group ( ^*∗*^*p* < 0.05). The level of CD8+ in the observation group was 22.84 ± 6.36, which was significantly lower than the control group ( ^*∗*^*p* < 0.05)**(**Figure 1**).**

### 3.4. Comparison of the Negative Emotional State of the Two Groups of Patients

After nursing, the SAS score and SDS score of the two groups were significantly decreased ( ^*∗*^*p* < 0.05), and the scores of the observation group were decreased more significantly (^Δ^*p* < 0.05), as shown in Table 4.

### 3.5. Comparison of the Quality-of-Life Scores between the Two Groups of Patients

Before nursing, there was no statistically significant difference in the quality-of-life scores between the two groups (*p* > 0.05). After nursing, the scores of the two groups of patients in terms of social/family status, physical function, physiological function, and emotional status were increased ( ^*∗*^*p* < 0.05), and the observation group was significantly higher than the control group (^Δ^*p* < 0.05) (Table 5).

### 3.6. Comparison of Tumor Marker Levels between the Two Groups of Patients

Before nursing, there was no significant difference in serum CA199 and CEA levels between the two groups of patients (*p* > 0.05). After nursing, the levels of tumor markers in the two groups were significantly decreased ( ^*##*^*p* < 0.01), and the observation group was downregulated more significantly than the control group (#*p* < 0.05) (Figures 2 and 3).

### 3.7. Comparison of the Two-Year Cumulative Survival Rate of the Two Groups of Patients

The two-year cumulative survival rate of the observation group was 78.18%, and the two-year cumulative survival rate of the control group was 54.55%. The observation group was significantly higher than the control group (*p* < 0.05) (Figure 4).

## 4. Discussion

Ovarian cancer is a malignant tumor with high clinical incidence [14]. With the improvement of people's living standards, women's pressure from work and life is increasing, coupled with environmental pollution and other factors, the incidence of ovarian cancer is increasing year by year, and the death rate is also increasing, which has been highly concerned by the medical community [15]. At present, there is no accurate and effective early diagnosis method for ovarian cancer, and it has progressed to the middle and late stage when it is diagnosed. Meanwhile, the treatment method is still based on traditional surgical resection, supplemented by radiotherapy and chemotherapy [16]. However, not only do patients have to suffer painful side effects during radiotherapy and chemotherapy, but also the rapid spread of tumor cells may lead to a high recurrence rate, which greatly reduces the patient's quality of life and life safety, bringing great trouble to the physical and mental health of patients [17]. As a treatment method that has been widely used in the treatment of ovarian cancer in recent years, traditional Chinese medicine (TCM) has the advantages of simple operation, less toxic side effects, and high security advantage. It can effectively control the development of the disease, alleviate the suffering of patients, and improve the quality of the patient's quality of life and survival. In clinical cancer treatment, it has been widely recognized by patients [18]. However, when patients with ovarian cancer learn that they have advanced cancer, they will generally experience nervousness, anxiety, denial, depression, and even resistance to treatment. At the same time, studies have confirmed that these negative psychological emotions can lead to a decrease in the immune function of patients with malignant tumors, which in turn will affect the treatment effect and quality of life of the patients [19]. Other studies have shown that ovarian cancer patients need to have a light diet and a reasonable diet control, and poor dietary habits will adversely affect the treatment of advanced ovarian cancer patients. Therefore, it is of great significance to improve the quality of life and prolong the survival time of ovarian cancer patients to pay attention to the changes of their psychological state and control their dietary habits while providing effective treatment for ovarian cancer patients [20]. Nursing should be based on the patient's condition and actual conditions, implement high-quality psychological interventions and high-quality diet care, and provide guidance on TCM, which reflects the comprehensiveness and individualization of the treatment process [21]. The implementation of psychological care for patients can improve patients' bad mood, promote their confidence in treatment, and improve treatment compliance, thereby enhancing the treatment effect.

This present study showed that the clinical efficacy of the observation group after nursing was significantly higher than that of the control group (*p* < 0.001), and the nursing satisfaction and treatment compliance of the observation group after nursing were significantly higher than that of the control group (*p* < 0.01), indicating that the nursing staff's practice of psychological intervention and dietary guidance for patients with advanced ovarian cancer provides positive psychological support to patients, establishes a good doctor-patient relationship with patients, strengthens patients' trust in medical staff, and is willing to actively cooperate with treatment, thereby improving clinical efficacy. Tumor markers are produced during the proliferation of tumor cells and are of great value for tumor diagnosis and prognosis. Meanwhile, the growth of malignant tumors has a greater relationship with the body's immune function. Immune function is an important indicator for evaluating the therapeutic effect of malignant tumors [22, 23]. The results of this study showed that 4 weeks after treatment, the CD3+, CD4+, CD4+/CD8+ levels in the observation group were higher than those in the control group (*p* < 0.05). The CD8+ level was lower than the control group (*p* < 0.05). The CA19-9 and CEA levels in the observation group were lower than the control group (*p* < 0.05), consistent with the results of studies reported by Hao et al. [24], suggesting that the prescription of tonifying kidney and removing blood stasis can disperse the masses and strengthen the body, clear heat and detoxify, invigorate the kidney, and replenish qi [25]. The prescriptions of *Astragalus*, *Codonopsis*, *Atractylodes*, and Poria have the functions of invigorating the spleen and qi, diuresis and swelling, and strengthening the body. ZZ nourishes the liver and kidney and can enhance the immune function against tumors. Taizishen can invigorate the spleen and stomach and improve immunity. Huangjing nourishes qi, replenish lung yin, and replenish kidney yin. Scrophulariaceae and *Scutellaria barbata* can detoxify, clear away heat and dispel blood stasis, nourish the yin, and cool the blood; *Gallus gallus domesticus* invigorates the spleen, eliminates food, and promotes dampness; Shansi mushroom dissipates nodules and eliminates carbuncle, clears heat, and detoxifies [26–30]. In modern pharmacology, the combination of various drugs can promote the body to secrete immune factors, reduce the level of tumor markers, and improve the therapeutic effect. The combined use of psychological intervention and dietary guidance can significantly improve the body's immune function and significantly reduce the level of tumor markers [31]. Results showed that the patients' negative emotions, such as depression and anxiety, were significantly improved after continuous psychological intervention in the observation group. Moreover, the functional status, physical status, emotional status, and social and family status scores in the observation group were significantly better than those of the control group. The two-year cumulative survival rate of the observation group was also significantly higher than that of the control group (*p* < 0.05), which further illustrates that the patients with advanced ovarian cancer who are treated with Bushen Quyu Decoction can be given continuous psychological intervention and reasonable dietary guidance, which can effectively eliminate the patient's negative emotions, such as anxiety and depression, effectively improve the patient's nursing effect, ultimately improve the patient's quality of life, and effectively extend the patient's survival time.

## 5. Conclusion

In summary, the Bushen Quyu Decoction combined with psychological intervention and diet guidance to treat patients with advanced ovarian cancer can effectively alleviate the patients' negative emotions, improve the patient's immune function, reduce the level of tumor markers, further improve the patient's quality of life and nursing satisfaction, improve the treatment effect, and promote the rehabilitation of patients; it is worthy of clinical application.

## Figures and Tables

**Figure 1:** Comparison of immune function between two groups after nursing. (a) Comparison of CD3+ level between the two groups. (b) Comparison of CD4+ level between the two groups. (b) Comparison of CD8+ level between the two groups. (b) Comparison of CD4+/CD8 level between the two groups. *∗p* < 0.05.

**Figure 2:** Comparison of serum CA199 levels between the two groups before and after nursing.

**Figure 3:** Comparison of serum CEA levels in the two groups before and after nursing.

**Figure 4:** Comparison of two-year cumulative survival rate between the two groups.

**Table 1:** Comparison of clinical efficacy between the two groups [n (%)].

Group	Cases	Complete remission	Partial remission	Stable	Progression	Total effective rate
Observation group	110	14 (12.73)	57 (51.82)	29 (26.36)	10 (9.09)	71 (64.55)
Control group	110	3 (2.73)	32 (29.09)	48 (43.64)	27 (24.54)	35 (31.82)
*χ* ^2^						26.639
*p*						<0.001

**Table 2:** Comparison of nursing satisfaction between the two groups [n (%)].

Group	Cases	Very satisfied	Relatively satisfied	Dissatisfied	Nursing satisfaction
Observation group	110	33	71	6	104 (94.55)
Control group	110	15	78	17	93 (84.55)
*p*					<0.01

**Table 3:** Comparison of treatment compliance between the two groups [n (%)].

Group	Cases	Full compliance	Partial compliance	Noncompliance	Compliance
Observation group	110	41	67	2	108 (98.18)
Control group	110	28	63	19	91 (82.73)
*p*					<0.001

**Table 4:** Comparison of negative emotional state between the two groups (*x* ± *s*).

Group	Cases	SAS scores		SDS scores	
		Before care	After care	Before care	After care
Observation group	110	72.56 ± 7.13	34.67 ± 5.23^∗△^	69.78 ± 7.65	37.66 ± 5.17^∗△^
Control group	110	71.42 ± 7.36	47.24 ± 6.71^∗^	70.54 ± 7.82	52.03 ± 6.21^∗^
*t*		0.362	11.423	0.278	13.754
*p*		>0.05	<0.05	>0.05	<0.05

**Table 5:** Comparison of quality-of-life scores between the two groups (*x* ± *s*).

Group	Cases		Social/family status	Physical function	Physiological function	Emotional status
Observation group	110	Before care	32.54 ± 3.66	28.97 ± 2.13	31.72 ± 3.75	29.61 ± 3.48
		After care	72.63 ± 4.47^∗△^	73.32 ± 5.96^∗△^	76.84 ± 4.21^∗△^	71.24 ± 5.33^∗△^
Control group	110	Before care	31.87 ± 3.72	29.46 ± 2.34	32.26 ± 3.41	28.77 ± 3.73
		After care	54.52 ± 6.13^∗^	56.26 ± 5.74^∗^	61.37 ± 5.42^∗^	57.12 ± 6.37^∗^
*t*			5.632	4.541	6.125	4.723
*p*			<0.05	<0.05	<0.05	<0.05

## Data Availability

The datasets used and/or analyzed during the present study are available from the corresponding author on reasonable request.
